This article has been retracted.

# Endogenous Urotensin II Selectively Modulates Erectile Function through eNOS

**DOI:** 10.1371/journal.pone.0031019

**Published:** 2012-02-02

**Authors:** Roberta d'Emmanuele di Villa Bianca, Emma Mitidieri, Ferdinando Fusco, Elena D'Aiuto, Paolo Grieco, Ettore Novellino, Ciro Imbimbo, Vincenzo Mirone, Giuseppe Cirino, Raffaella Sorrentino

**Affiliations:** 1 Interdepartmental Research Centre for Sexual Medicine (CIRMS), University of Naples, Federico II, Naples, Italy; 2 Department of Experimental Pharmacology, University of Naples, Federico II, Naples, Italy; 3 Section of Clinical Immunology, Department of Clinical and Experimental Medicine, Second University of Naples, Naples, Italy; 4 Department of Pharmaceutical and Toxicological Chemistry, University of Naples, Federico II, Naples, Italy; University of Illinois at Chicago, United States of America

## Abstract

**Background:**

Urotensin II (U-II) is a cyclic peptide originally isolated from the neurosecretory system of the teleost fish and subsequently found in other species, including man. U-II was identified as the natural ligand of a G-protein coupled receptor, namely UT receptor. U-II and UT receptor are expressed in a variety of peripheral organs and especially in cardiovascular tissue. Recent evidence indicates the involvement of U-II/UT pathway in penile function in human, but the molecular mechanism is still unclear. On these bases the aim of this study is to investigate the mechanism(s) of U-II-induced relaxation in human corpus cavernosum and its relationship with L-arginine/Nitric oxide (NO) pathway.

**Methodology/Principal Findings:**

Human corpus cavernosum tissue was obtained following in male-to-female transsexuals undergoing surgical procedure for sex reassignment. Quantitative RT-PCR clearly demonstrated the U-II expression in human corpus cavernosum. U-II (0.1 nM–10 µM) challenge in human corpus cavernosum induced a significant increase in NO production as revealed by fluorometric analysis. NO generation was coupled to a marked increase in the ratio eNOS phosphorilated/eNOS as determined by western blot analysis. A functional study in human corpus cavernosum strips was performed to asses eNOS involvement in U-II-induced relaxation by using a pharmacological modulation. Pre-treatment with both wortmannin or geldanamycinin (inhibitors of eNOS phosphorylation and heath shock protein 90 recruitment, respectively) significantly reduced U-II-induced relaxation (0.1 nM–10 µM) in human corpus cavernosum strips. Finally, a co-immunoprecipitation study demonstrated that UT receptor and eNOS co-immunoprecipitate following U-II challenge of human corpus cavernosum tissue.

**Conclusion/Significance:**

U-II is endogenously synthesized and locally released in human corpus cavernosum. U-II elicited penile erection through eNOS activation. Thus, U-II/UT pathway may represent a novel therapeutical target in erectile dysfunction.

## Introduction

Urotensin II (U-II) is a cyclic peptide hormone derived from pre-pro-U-II by urotensin-converting enzyme. It was first isolated from teleost fish and homologues subsequently were identified across the evolutionary spectrum, including mammals and man. U-II causes both vasoconstriction and vasodilation depending by the vascular district and the species considered [1]–[6]. Its vasoactive effect is mediated by binding to a GPR14 (UT receptor), a G protein-coupled receptor [7]. U-II is secreted from heart and several other tissues into the circulation [8]. However, the source of U-II production in the human body remains to be elucidated. Both U-II and UT receptor are expressed widely within the cardiovascular system, and their expression is up-regulated in human cardiovascular disease, including congestive heart failure, hypertension, type II diabetes and diabetic nephropathy [9]–[11]. Collectively, these data indicate U-II as potential modulator of cardiovascular homeostasis in human.

Recently, we have demonstrated the involvement of U-II/UT pathway in erectile function [12]. Indeed, an intra-cavernous injection of U-II in rats causes an increase in intra-cavernous pressure without affecting systemic blood pressure. It has also been demonstrated that UT receptor is present in human corpus cavernosum (HCC). It is located on the endothelium and it mediates an endothelium-dependent relaxation involving the L-arginine/nitric oxide (NO) pathway [12]. It is well established that the L-arginine/NO pathway plays a major role in erectile function in man [13], [14]. NO is produced by a group of enzymes called nitric oxide synthase (NOS) that by converting L-arginine into L-citrulline produce NO [15], [16]. The endothelial NOS (eNOS) is constitutively expressed within the vascular system, it is tightly regulated and produces physiologically relevant levels of NO.

The regulation of eNOS involves multiple molecular mechanisms that act in concert to both positively or negatively affect the function of this enzyme. eNOS is classified as a constitutive and strictly calcium/calmodulin-dependent enzyme [17]. The calcium levels as well as the heath shock protein 90 (Hsp90) recruitment increase the catalytic activity of eNOS [18], [19]. The eNOS-associated Hsp90 may also serve as a scaffolding protein, facilitating the organization of additional associated regulatory proteins. In addition, fluid shear stress or other stimuli by phosphorylation can shift eNOS to an higher state of activation [20]. For example, bradykinin enhances eNOS phosphorylation; this effect is maximal after 5 minutes and it is maintained for at least 20 minutes in cultured endothelial cells [21]. In recent years, it has been reported that eNOS phosphorylation at serine^1177^ by phosphatydilinositol 3 kinase (PI3K)/protein kinase B (Akt) is critical for the maintenance of full penile erection [22], [23]. Thus eNOS activity is finely regulated and can shift to an higher degree of activation following molecular modulation [17]–[23].

The present study investigates the relationship between U-II/UT and L-arginine/NO pathway in human corpus cavernosum. Our data demonstrate that U-II pro-erectile response relies on eNOS-derived NO, contributing to the maintenance of full penile erection.

## Results

### U-II is present as mRNA in HCC

The RT-PCR analysis (Figure 1) clearly demonstrated the U-II presence in HCC samples. Since it has been reported that U-II is over-expressed in human tumoural cell lines SW-13 [24], a positive control by using SW-13 cells was performed, too. No amplifications were observed when PCR was performed in same conditions but without cDNA.

**Figure 1:** Quantitative RT-PCR for U-II in HCC. U-II is expressed as mRNA in HCC samples. Human tumoural cells SW-13 were used as positive control. Data were normalized on the basis of GAPDH and expressed as mean ± standard error of the mean (SEM) of three different human specimens.

Taken together, these data demonstrate that U-II can be locally synthesized and endogenously released in HCC.

### U-II vasorelaxant effect involves eNOS activation

As previously described U-II causes an endothelium- and NO-dependent relaxation in pre-contracted HCC strips [12]. A pharmacological eNOS modulation was operated by using inhibitors that either interfere with Hsp90 recruitment (geldanimycin) or inhibit phosphorylation (wortmannin). Both wortmannin (0.1 µM) or geldanamycin (1 µM) significantly reduced U-II induced relaxation of human tissues (Figure 2 A, ***p<0.001 and **p<0.01).

**Figure 2:** Panel A: U-II induced concentration-response curve (0.1 nM–10 µM) in HCC strips was significantly inhibited by pre-treatment with wortmannin (0.1 µM), PI3K inhibitor, or geldanamycin (1 µM) Hsp90 inhibitor (***p<0.001 and ** p<0.01 *versus* vehicle). Data were expressed as the mean ± standard error of the mean (SEM) of six different specimens. Data were analyzed by ANOVA followed by Bonferroni post test. Panel B: NOx (total nitrite) production in HCC tissue incubated with U-II (1 nM-10 µM) or vehicle for 30 min. U-II caused a significant increase in NO production compared with vehicle (*p<0.05, **p<0.01, ***p<0.001). Data were expressed as mean ± standard error of the mean (SEM) from four different specimens and analyzed by ANOVA followed by Bonferroni post test.

### U-II promotes NO production in HCC

In order to confirm the NO involvement in U-II/UT signaling we evaluated the NO production in HCC homogenate tissues stimulated with U-II (1 nM–10 µM). Data, expressed as total nitrite, clearly showed that U-II caused a significant increase in NOx production compared with vehicle (Figure 2 B, *p<0.05, **p<0.01, ***p<0.001).

### U-II induces eNOS phosphorylation in HCC

To further asses the U-II involvement in eNOS activation we performed a western blot study. The protein expression of eNOS as well as phosphorylated eNOS^Ser 1177^ (p-eNOS) in tissues incubated with U-II (10 µM), at scheduled time, was evaluated. U-II induced eNOS phosphorylation in a time-dependent manner, reaching its maximum at 30 minutes (Figure 3 A, *p<0.05). Thus 30 minutes of incubation has been chosen as the time point to perform the experiments by using inhibitors. Wortmaninn (0.1 µM), an irreversible inhibitor of PI3K, but not geldamycin, reverted significantly eNOS phosphorylation induced by U-II challenge (***p<0.001, Figure 3 B).

**Figure 3:** Western blot analysis for eNOS and p-eNOS^Ser-1177^ in HCC tissue. Panel A: U-II (10 µM) caused an increase in eNOS phosphorylation expressed as p-eNOS/eNOS ratio in a time-dependent manner (*p<0.05 *vs* vehicle). Panel B: U-II-induced eNOS phosphorylation (**p<0.01 *vs* vehicle), was significantly reverted by wortmannin (0.1 µM), PI3K inhibitor, (°p<0.05 *vs* U-II) but not by geldanamicin (1 µM), Hsp90 inhibitor. Data were expressed as the mean ± standard error of the mean (SEM) of four different specimens and were analyzed by ANOVA followed by Bonferroni post test.

### U-II induces the recruitment of eNOS to UT receptor in HCC

The co-immunoprecipation assay allows to identify protein-protein/enzyme interaction. Thus, to confirm the relation between U-II/UT pathway and eNOS, we performed the eNOS precipitation and monitored the co-precipitation of UT receptor in HCC tissues incubated for 30 minutes with U-II (10 µM) or vehicle. U-II induced the formation of the immunocomplex between UT and eNOS (Figure 4).

**Figure 4:** Co-immunoprecipitation analysis of UT receptor and eNOS. Tissues were stimulated with either vehicle (A) or U-II (C), lysates were incubated with mouse anti-eNOS. Lanes B and D correspond to the negative control of A and C, respectively. The western blot was probed with rabbit anti-GPR14 (UT receptor). U-II but not vehicle caused the co-immunoprecipation between eNOS and UT receptor.

## Discussion

Human penile erection is a resultant of several complex mechanisms. A key issue is the balance between contracting and relaxant factors which are instrumental in order to achieve penile erection. It is now well accepted that NO plays a major role in induction and maintenance of erection [25]–[28]. Recently we have reported that U-II-induced relaxation in HCC is endothelium- and NO-dependent [12]. On this basis we have proposed that U-II, physiologically circulating in our body [8], contributes to penile homeostasis. Our present finding further extends the importance of this signaling pathway and confirms that endothelium is necessary.

We have demonstrated that mRNA for U-II is present in the human tissue. This finding indicates that U-II can be locally endogenously synthesized within the HCC and that U-II/UT pathway is involved within erection physiology. The exclusive presence of UT receptor on the endothelial cells in human penile tissue [12] further corroborates this concept. Based on this and our previous finding, we have hypothesized an interaction between UT receptor and eNOS at molecular level within the endothelium. Following this hypothesis we performed a co-immunoprecipitation study. The formation of the immunocomplex demonstrated that a link exists between eNOS and U-II/UT pathway within the human penile tissue. This molecular evidence was functionally confirmed. Indeed, the incubation of HCC homogenates with U-II caused a concentration-dependent increase in NOx production. Interestingly, the highest U-II concentration elicited a six fold increase in NOx generation. Thus, U-II released within the corpus cavernosum binds its receptor on endothelial cells leading to eNOS activation and in turn to NO production. Basically, U-II-induced relaxation contributes to eNOS-derived NO generation in HCC. But how activation of this pathway leads to an increase production of eNOS-derived NO? To date it is well consolidate the concept that neuronal NOS (nNOS) and eNOS mediate the initiation and maintenance of penile erection, respectively [22]. Neuronal signal initiates penile erection by activating nNOS that elicits a rapid and transient NO release causing an increase in blood flow [29]. The resulting shear stress force on the endothelium activates the PI3K/Akt/eNOS phosphorylation cascade, causing more sustained NO release and relaxation [22], [30]. Indeed, Akt-phoshorylated eNOS results 15 to 20 fold more active that un-phospohorylated eNOS [31]. In other words, the phosphorylation of eNOS shifts the enzyme at higher state of activation, boosting NO production [32].

In the human body, the penis is one of the organ physiologically subjected to shear stress and the resultant eNOS phosphorylation^Ser1177^ plays a key role in the maintenance of full penile erection [22]. Therefore, we performed a pharmacological modulation of the eNOS phosphorylation in order to investigate if U-II activity relies on this mechanism. U-II caused a significant increase in eNOS phosphorylation ^Ser1177^ in a time-dependent manner. The irreversible inhibition of PI3K/Akt operated by wortmannin, reverted the phosphorylation induced by U-II. Also in this case the molecular finding has been confirmed through a functional study. Indeed, U-II relaxant effect on HCC was virtually abolished by wortmannin.

Another recognized key player in the mechanism of eNOS activation is Hsp90. In fact, shear stress as well as some other endogenous substances enhances the interaction between Hsp90 and eNOS [18], [19]. The increased association of eNOS to Hsp90 shifts the enzyme to an higher active state, too. Basically, Hsp90 acts as an allosteric modulator of eNOS by inducing conformational changes in the enzyme that result in an increased activity [33]. Geldanamycin, an Hsp 90 inhibitor, blocked U-II induced relaxation of HCC strips at the same extent of wortmannin. Experimental evidence suggests that Hsp90-eNOS hetero-complex occurs simultaneously with other signaling events such as the mobilization of intracellular calcium and/or protein phosphorylation [34]. Therefore, it appears feasible the U-II/UT pathway contributes to the maintenance rather than triggering erection. Indeed, the pro-erectile effect of U-II is strictly dependent upon eNOS derived-NO generation. The obligatory role for eNOS-derived NO in U-II effect is supported by the finding that i) blockade of eNOS phosphorylation and Hsp90 coupling abrogates U-II effect ii) incubation of HCC tissue with U-II causes a notable increase in NO generation.

In conclusion , U-II/UT pathway contributes to the physiology of erection through eNOS-derived NO. UII/UT pathway once activated, most likely by the shear stress due to the erection, causes eNOS phosphorylation and Hsp90 recruitment shifting eNOS activity to a more activate state. This in turn leads to a sustained NO release which contribute to the maintenance of the ongoing erection.

Thus, U-II/UT pathway could represent an important novel target in order to find new pharmacological approaches in erectile dysfunction. Indeed, it is known that a certain percent of patients (about 35%) do not respond to PDE5 inhibitors [35]. As PDE5 inhibitors and U-II share the same target NO, it is plausible that in the next future U-II agonists might be used in combination with PDE5 inhibitors in order to enhance cGMP signaling. Indeed, it could be that in some cases there is only a limited amount of endothelium functionally working and the PDE5 inhibition by itself will not be sufficient to sustain the erection triggered. In this case the combination with the UII agonist could exert a synergistic effect.

## Methods

### Peptide

The human U-II was synthesized and purified at the Department of Pharmaceutical and Toxicological Chemistry of the University of Naples, Federico II. The peptide was obtained by solid-phase peptide synthesis as previously reported [36]. Purification was achieved using a semi-preparative reversed phase high-performance liquid chromatography (HPLC) C18 bonded silica column (Vydac 218TP1010; The Separations Group Inc., Hesperia, CA, USA). The purified peptide was 99% pure as determined by analytical reversed-phase HPLC. The correct molecular weight were confirmed by mass spectrometry and amino acid analysis.

### Human Tissue

In male-to-female transsexuals undergoing surgical procedure for sex reassignment, the penis and testicles were amputated and a neo-vagina was created to simulate female external genitalia. All the surgical procedures were performed at the Department of Urology, University of Naples, Federico II, Naples, Italy [37]. The corpora cavernosa were carefully excised from the penis immediately after amputation and placed in ice-cold oxygenated Krebs' solution [37]. All patients were informed of all procedures and gave their written consent. Local Ethical Committee (Faculty of Medicine and Surgery; University of Naples Federico II, via Pansini, 5; 80131, Naples, Italy) approved the use of human corpus cavernosum tissue for in vitro studies.

### Real-Time Quantitative Reverse Transcriptase Polymerase Chain Reaction (RT-PCR)

The presence of U-II was determined by quantitative PCR. Briefly, total RNA from omogenated HCC tissue was extracted by using TRIzol reagent (Invitrogen, Milan, Italy), to eliminate genomic DNA contamination 1 µg of above RNA was treated with RQ1 RNase-free DNase I (Promega Corporation, Madison, USA), according to the manufacturer's recommendations. Reverse transcription was performed using M-MLV Reverse Transcriptase (Invitrogen, Milan, Italy) according to the manufacturer's recommendations, and 20 ng of cDNA samples were used for quantitative PCR. Samples were run in triplicate in 25-µL reactions using an 7500 Real Time PCR System (Applied Biosystems, Foster City, CA). Amplification was done using Sybr Green PCR Master Mix (Applied Biosystems, Monza, Italy). U-II-specific forward primers 5′-GCACTGTTTGCTTTGGACTCC-3′and reverse primer : 5′-TGGTCGTCCATGCACAGATT-3′, and human GAPDH forward primer 5′-AACGGATTTGGTCGTATTGGGC- 3′ and reverse primer 5′-TCGCTCCTGGAAGATGGTGATG-3′ were specifically designed using Primer Express Software 2.0 and validated for their specificity. Samples were incubated at 50°C for 2 min and at 95°C for 10 min followed by 40 cycles at 95°C for 15 s and 60°C for 1 min. Differences in cDNA input were corrected by normalizing signals obtained with primers specific for glyceraldehydes-3-phosphate dehydrogenase (GAPDH). To exclude nonspecific amplification and/or the formation of primer dimers, control reactions were performed in the absence of target cDNA. In order to validate the results we used human tumoural cell lines SW-13 as positive control [24]. Gene expression levels were calculated using the 2^−ΔCT^ method and are presented as ratio between mean fold change of target gene and GAPDH ± standard error. Data were expressed as mean ± standard error of the mean (SEM) from three different specimens.

### NOx determination

HCC tissues were incubated with U-II at different concentration (1 nM–10 µM) or vehicle for 30 minutes at 37°C. The reaction was stopped in liquid nitrogen. Homogenate tissues were incubated in a microplate with cadmium (50 mg/well) for 1 h to convert the inorganic anions nitrate (NO_3_) to nitrite (NO_2_). After centrifugation at 14,000 rpm for 15 min, total nitrite (NOx) content was determined fluorometrically in microtiter plates (PerkinElmer Instruments, LS55; UK) using a standard curve of sodium nitrite [38]. NOx content was calculated by using the internal standard curve. Data were expressed as mean ± standard error of the mean (SEM) from four different specimens and analyzed by using analysis of variance (ANOVA) followed by Bonferroni post hoc test. The level of statistical significance was taken as *p*<0.05.

### Functional reactivity of HCC Strips

Longitudinal strips (2 cm) of HCC were dissected and isolated from the trabecular structure of the penis [25]. Krebs' solution had the following composition (mM): 115.3 NaCl; 4.9 KCl; 1.46 CaCl_2_; 1.2 MgSO_4_; 1.2 KH_2_PO_4_; 25.0 NaHCO_3_; 11.1 glucose (Carlo Erba, Milan, Italy). HCC strips were mounted in organ bath containing oxygenated (95% O_2_ and 5% CO_2_) Krebs' solution at 37°C. HCC strips were connected to isometric force-displacement transducers (model 7002, Ugo Basile, Comerio, Italy) and changes in tension were recorded continuously by using a software (Datacapsule, Basile, Comerio, Italy). Tissues were preloaded with 2 g of tension and allowed to equilibrate for 90 minutes in Krebs' solution. After equilibration, tissues were standardized by performing repeated phenylephrine (PE; 3 µM; Sigma, Milan, Italy) contractions until three equal responses were obtained. Endothelial integrity was assessed by using acetylcholine (Ach; 0.01–10 µM; Sigma, Milan, Italy) and tissues that showed a relaxation effect less that 80% were discarded. A concentration response curve to U-II (0.1 nM–10 µM) was obtained in the presence of endothelium, using HCC strips pre-contracted with PE (3 µM). In order, to investigate the involvement of L-arginine/NO pathway in U-II-induced relaxation we operated a pharmacological modulation. HCC strips were incubated for 30 minutes with either wortmannin (0.1 µM, Tocris, UK) an irreversible inhibitor of PI3K or geldanamycin (1 µM, Sigma, Milan, Italy) an Hsp90 inhibitor before U-II challenge. The doses of wortmannin (0.1 µM) and geldamycin (1 µM) were selected by a preliminary dose-finding study (data not shown).

Data were calculated as % of relaxation to PE tone and expressed as the mean ± standard error of the mean (SEM) of six different specimens. The results were analyzed by using analysis of variance (ANOVA) followed by Bonferroni post hoc test. The level of statistical significance was taken as *p*<0.05.

### Western Blot Analysis

In order to evaluate the effect of U-II on the eNOS phopsphorylation -Ser 1177 (p-eNOS ^Ser 1177^), HCC tissues were incubated with the peptide (10 µM) at scheduled time (5, 15, 30 and 60 minutes). In another set of experiments, tissues were pre-treated with wortmannin (0.1 µM, Tocris, UK) or geldamycin (1 µM, Sigma, Milan, Italy) and thereafter incubated with U-II (10 µM) or vehicle for 30 minutes. Next, HCC tissues were homogenized in modified RIPA buffer (Tris-HCl 50 mM, pH 7.4, Triton 1%, sodium deoxycholate 0.25%, NaCl 150 mM, ethylenediaminetetraacetic acid 1 mM, phenylmethylsulphonyl fluoride 1 mM, aprotinin 10 µg/mL, leupeptin 20 µM, NaF 1 µM, sodium orthovanadate 1 µM) by liquid nitrogen. Protein concentration was estimated by the Bio-Rad protein assay using bovine serum albumin (BSA) as standard. Equal amounts of protein (50 µg) of the tissue lysates were separated on 8% sodium dodecyl sulfate polyacrylamide gels and transferred to a polyvinylidene fluoride membrane. Membranes were blocked by incubation in phosphate-buffered saline (PBS) containing 0.1% v/v Tween 20, non fat dry milk (5%) and NaF (50 mM) for 1 hours, followed by overnight incubation at 4°C with rabbit anti-p-eNOS^Ser-1177^ polyclonal antibody (1∶1000, Cell Signaling, DBA, Italy) and with mouse eNOS monoclonal antibody (1∶1000; BD Transduction Laboratories). The filters were washed extensively in PBS containing 0.1% v/v Tween 20, before incubation for 2 hours with horseradish peroxidase-conjugate anti rabbit secondary antibody (1∶5000). Membranes were then washed and developed using enhanced chemiluminescence substrate (Amersham Pharmacia Biotech, San Diego, CA, USA). The data were evaluated by densitometric analysis and expressed as p-eNOS/eNOS ratio.

Data were expressed as mean ± standard error of the mean (SEM) of four different specimens. The results were analyzed by using analysis of variance (ANOVA) followed by Bonferroni post hoc test. The level of statistical significance was taken as *p*<0.05.

### UT receptor and eNOS co-immunoprecipitation

HCC samples were homogenized (500 µg) and incubated with 20 µl of Protein A–coupled sepharose beads and 1 µg/ml of IgG mouse at 4°C for 3 h. The samples were centrifuged (600 rpm for 15 sec) and the supernatants were incubated overnight at 4°C with 20 µl of mouse eNOS monoclonal antibody (Cell Signaling, DBA, Milan, Italy) or normal mouse serum (to evaluate non-specific binding) on a rotating wheel.Next, the samples were incubated with 40 µl of Protein A–coupled sepharose beads at 4°C for 2 h and centrifuged (600 rpm for 15 sec). The pellets were extensively washed and then suspended in 3× Laemmly buffer. After heating at 95°C for 5 minutes, samples were subjected to Western blot analysis developed for UT (1∶1000; GPR14 (H-90), Santa Cruz Biotechnology Inc., Heidelberg, Germany).
